The article "Effects of Nalbuphine Combined with Anterior Serratus Plane Block in Elderly Patients Undergoing Thoracoscopic Surgery" was published in 2022. Journal: J Healthc Eng.

# Effects of Nalbuphine Combined with Anterior Serratus Plane Block in Elderly Patients Undergoing Thoracoscopic Surgery

**DOI:** 10.1155/2022/7408951

**Published:** 2022-02-10

**Authors:** Ying Liu, Yunpeng Li, Chao Wu, Hang Li

**Affiliations:** ^1^Department of Anesthesiology, Dongyang People's Hospital, Zhejiang Province, Dongyang 322100, Zhejiang, China; ^2^Department of Ultrasound, Dongyang People's Hospital, Zhejiang Province, Dongyang 322100, Zhejiang, China

## Abstract

Postoperative pain in elderly patients with lung cancer after thoracoscopic surgery is still an important factor affecting the prognosis of patients. In this study, 200 elderly patients with lung cancer who were positive and planned to undergo video-assisted thoracoscopic surgery were randomly divided into four groups: control group, SAPB (serratus anterior plane block) group, Nalbuphine group and Nalbuphine + SAPB group. The effects of drugs and nerve block on the perioperative indexes of elderly patients were observed. The results showed that ① The VAS and SAS scores of postoperative analgesia in the Nalbuphine + SAPB group were lower than those in the single group and the control group. ② The postoperative spontaneous respiratory recovery time, extubation time, resuscitation room stay time, extubation cough, restlessness and respiratory depression in the Nalbuphine + SAPB group were lower than those in the single group and the control group. ③ The heart rate (HR), systolic blood pressure (SBP), diastolic blood pressure (DBP), mean arterial pressure (MAP) and blood oxygen saturation (SpO2) of patients in Nalbuphine + SAPB group before induction, T2 after intubation, T3 before skin incision, T4 after skin incision, T5 after chest closure and T6 after extubation were lower than those in single group and control group. Therefore, this study concluded that Nabufine combined with SAPB can make the vital signs of intraoperative patients more stable, which is worthy of clinical promotion.

## 1. Introduction

VATS (Video-assisted thoracoscopic operation) has grown gradually and allows mediastinal tumor resection and wedge resection. Widespread utilization of modern VATS provide postoperative retrieval of the lungs. The VATS also potentially decreases cost, operative trauma, and allows earlier ambulation. The pain experienced is normally average and is mostly pain at the incision in the chest tube site, elastic tissues and intercostal muscles. Over-all management of Nalbuphine analgesia treatment, that is widely the core of pain monitor procedures, may involve intravenous opioids regional blocks and oral non-steroidal anti-seditious medicines [1]. Perfect Nalbuphine treatment offers effectual pain assistance, lessens side effects, and augments patient comfort. With progress in ultrasonic technology, regional block technologies happen to be more popular and involve erector spinal block, as well as thoracic epidural block (TEB). TEB is a technique in which analgesia is produced by injecting local anesthetic agent by itself or combined with additives or alone into the epidural space. TEB is presently the best paradigm for Nalbuphine treatment in thoracic operation, though it needs usual coagulation work, and the letdown rate in medical work is up to 29 percent because of problematic catheter detachment and catheterization.

The article "Effects of Nalbuphine Combined with Anterior Serratus Plane Block in Elderly Patients Undergoing Thoracoscopic Surgery" was published in 2022. Journal: J Healthc Eng.

Furthermore, extreme epidural anesthesia (Nalbuphine) simply results to hypotension necessitating fluid change and possibly administration of vasoactive medicines that may result to the damage of microcirculation, in order to reinstate hemodynamic strength. Wang et al [2] adds that other probable extreme outcomes include pruritus, nausea, and vomiting, maybe due to the epidural opioids administration. In relieving thoracic pains, paravertebral can work well but needs many injections, spinal cord or nerve injury pneumothorax and this potentially increases the dangers of an overdose of local anesthetics. Ultimately, erector spinae block usually employed for the cure of chest pains at the posterior, has painful implications on post-operation stage of the anterolateral and lateral chest walls. SAPB is a new chest slab methodology started in 2013. SAPB is a local block initially established for analgesia after breast operation, and more recently as Nalbuphine treatment particularly for the elderly undergoing thoracoscopic surgery. Serratus plane block is a simple, effective and safe thoracic fascial plane block. SAPB process depends on the presence of two possible gaps on the face on the anterior of the serratus tissues or muscles, a deep muscle plane between the anterior regions of the serratus and the intercostal muscles, and the latissimus dorsi [3]. Nalbuphine is injected at the block of the two planes, hence alleviating pain at the chest walls [4]. The aim of the SABP is on the T9 and T2 intercostal branches at the nerve system to augment Nalbuphine at the posterior chest walls. VATs are steadily adopting this technique, though there are a few yet randomized managed testing to back its utilization in this situation [5]. At present, the thoracoscopic surgery makes a comparison of the time, mostly within a period of 48 hours postoperatively to the overview of the analog pain notch (VAS) ≥4.01 between local infiltration Nalbuphine treatment and SABP. This is mostly among the elderly persons undergoing VATS for lung malignance to see how it affects them over a specific period. This aids in correlating the usage of postoperative Nalbuphine treatment among the elderly patients. This is particularly crucial in ascertaining the SAPB in combination with Nalbuphine treatment in offering more safeguards among the elderly patients undergoing thoracoscopic surgery.

The article "Effects of Nalbuphine Combined with Anterior Serratus Plane Block in Elderly Patients Undergoing Thoracoscopic Surgery" was published in 2022. Journal: J Healthc Eng.

## 2. Methods

### 2.1. Subject- Elderly Patients

This research was done conforming to the Helsinki Declaration for research encompassing human subjects. All the elderly patients gave written informed consent to back their participation in this research. This research was undertaken with full consent from the Chinese Clinical Trial Registry way before enrolling the elderly patients to participate in this research.

### 2.2. Setting and Study Design

The elderly patients were put in the control group, SAPB group, Nalbuphine group and Nalbuphine + SAPB group through an arbitrary minute table, as well the group work kept in a closed wrapper, referred just to the doctors doing the nerve block surgeries [6]. The grouping of the patients was based on the simple randomization. The surgeons and elderly patients undergoing the intraoperative anesthesia (local Nalbuphine treatment) procedure, as well as the doctors doing postoperative pain, and valuations were unaware of the task assignments, as they were not opened and the lumps were done away from the operating theater. ① Control group (routine) regimen: midazolam 0.08mg/kg, sufentanil 0.4ug/kg, etomidate 0.3mg/kg, vecuronium 0.1mg/kg, propofol 6mg/kg/h, remifentanil 8ug/kg/h, 30min before suture, sufentanil 0.1ug/kg for analgesia during operation. ② SAPB group: midazolam 0.08mg/kg, sufentanil 0.4ug/kg, etomidate 0.3mg/kg, vecuronium 0.1mg/kg, SAPB after induction, propofol 6mg/kg/h, remifentanil 8ug/kg/h, 30min before suture, sufentanil 0.1ug/kg for analgesia during operation. ③ Nalbuphine group: midazolam 0.08mg/kg, sufentanil 0.4ug/kg, etomidate 0.3mg/kg, vecuronium 0.1mg/kg, propofol 6mg/kg/h and remifentanil 8ug/kg/h were used during operation. Before anesthesia induction, Nalbuphine 0.2mg/kg was given to relieve pain. ④ Nalbuphine + SAPB group: midazolam 0.08mg/kg, sufentanil 0.4ug/kg, etomidate 0.3mg/kg, vecuronium 0.1mg/kg, SAPB was performed after induction, propofol 6mg/kg/h and remifentanil 8ug/kg/h were used during operation, and nalbuphine 0.2mg/kg was given before anesthesia induction. Keep the perioperative heart rate and blood pressure in the normal range. If the blood pressure and heart rate rise or decrease by 30% in the basic value, give the corresponding vasoactive drugs for treatment; if the hemoglobin is lower than 100g/L, blood transfusion products should be selected according to the actual situation.

The article "Effects of Nalbuphine Combined with Anterior Serratus Plane Block in Elderly Patients Undergoing Thoracoscopic Surgery" was published in 2022. Journal: J Healthc Eng.

### 2.3. Main Research Indicators

The main indicators were heart rate (HR), systolic blood pressure (SBP), diastolic blood pressure (DBP), mean arterial pressure (MAP), and blood oxygen saturation (SPO_2_) in patients T1 before induction, T2 after intubation, T3 before skin incision, T4 after skin incision, T5 after chest closure, and T6 after extubation. The time of recovery when it comes to impulsive breathing, residence time in the resuscitation room, extubation time, the frequency of extubation choking, respiratory depression and agitation. The SpO2 a lesser amount of 90% for 15s or the rate of respiration less than 12 times for a period of 10 minutes. The VAS score was recorded before the onset of the operation, instantaneously after 4 hours, 8 hours, 12 hours, and 24 hours after extubation. Additionally, we compared the adverse events in the present study, and the adverse events were defied as the vomiting and nausea.

### 2.4. Statistical Analysis

The research examined quantitative data of abnormal or normal distribution with Mann–Whitney or t-test. This qualitative data was made in comparison to the set data utilizing Fisher's exact trial or *χ*^2^ test. Additionally, the assessing of the occasion-time data was with record-position test and curve of Kaplan-Meier.

### 2.5. Sample Size

In this study, 200 elderly patients with lung cancer who were positive and planned to undergo video-assisted thoracoscopic surgery were randomly divided into four groups: control group, SAPB group, Nalbuphine group and Nalbuphine + SAPB group. The effects of drugs and nerve block on the perioperative indexes of elderly patients were observed. The sample size for this research was 200 elderly patients. The main pointer was the period to VAS count four through the first two days post-operation. The valued median period following surgery to the first VAS count of four was 4 hours (SD = 9.3401) with indigenous Nalbuphine permeation in thoracoscopic operation. In theory the fruitful SAPB lasts for 12 hours (91% power and a 6% importance degree), which would need 50 elderly patients per unit. To report for lost patient figures, there was a composition of 20 patients in each unit.

## 3. Results

There were around 200 elderly patients qualified for the research, of which 80 were left out (40 did not endorse informed consent, 28 elderly patients had a history of chest surgeries, and 9 of the elderly patients were using Nalbuphine drugs. Whilst 3 of the elderly patients had difficulties with language expression).  Figure 1 is the flow chart of the study.

As articulated earlier, the main indicators were heart rate (HR), systolic blood pressure (SBP), diastolic blood pressure (DBP), mean arterial pressure (MAP), and blood oxygen saturation (Sp02) in patients T1 before induction, T2 after intubation, T3 before skin incision, T4 after skin incision, T5 after chest closure, and T6 after extubation. The elderly patients were presented with hypoxaemia, for managing severe respiratory distress. Ninety percent Sp02 to manage shock, through titrating to Sp02 ≥ 90% as well as initiating oxygen therapy at 5 L/min and titrate to SpO2. Cardiac output and oxygen consumption (VO2) measurements were affected through utilizing a CPX/D Medical Graphics metabolic analyzer. The determination of cardiac output was after 6 hours through employing the ancillary CO2 rebreathing technique. The data and statistical data encompassed the analysis of variance with repeated measures, that indicates that at the 6 hours, there was increased heart rate (HR) due to increase in metabolism, that resulted to a rise in VO2. The rise was occasioned by the HR (heart rate) response and the fall in SVR (systemic vascular resistance). The SBP (systolic blood pressure) and MAP (Mean arterial pressure) decreased while on the other hand there was increase in blood oxygen saturation. There were no major variations in the T2 after intubation, and skin incision. However, T5 after chest closure and extubation was vital in increasing metabolism during the thoracoscopic surgery.

The article "Effects of Nalbuphine Combined with Anterior Serratus Plane Block in Elderly Patients Undergoing Thoracoscopic Surgery" was published in 2022. Journal: J Healthc Eng.

There were no significant differences in terms of sex, BMI, or the time of operation (p > 0.05 in Table 1). The projected median period following the thoracoscopic surgery to the initial point VAS count was 5 hours (1.45 to 7.75) in the set of control and 12 h (7.45 to 16.35) in the SAPB set (log order test) (survival curve study): *P* = 0.009, suggesting protracted lasting postoperative Nalbuphine with ultrasound-led SAPB in comparison to indigenous infiltration Nalbuphine.

The number of elderly patients necessitating additional Nalbuphine at 7 hrs and 12 hrs after thoracoscopic operation was marginally greater(Table 2) (*P* < 0.05) in the set of control versus the set of SAPB, but there was no major variance among the sets in Nalbuphine prerequisite after the 12 hrs. There was no major variation among the sets in the dosage after interoperation of propofol and remifentanil (Table 3) (*P* > 0.05) or in the prevalence of post-operation vomiting as well as nausea (Table 4) (*P* > 0.05).

The postoperative spontaneous respiratory recovery time, extubation time, resuscitation room stay time and the incidence of extubation cough, restlessness and respiratory depression in the Nalbuphine + SAPB group were lower than those in the single group and the control group (Table 5)(*P < *0.05).

The article "Effects of Nalbuphine Combined with Anterior Serratus Plane Block in Elderly Patients Undergoing Thoracoscopic Surgery" was published in 2022. Journal: J Healthc Eng.

The heart rate (HR), systolic blood pressure (SBP), diastolic blood pressure (DBP), mean arterial pressure (MAP) and blood oxygen saturation (SpO2) of patients in Nalbuphine + SAPB group before induction, T2 after intubation, T3 before skin incision, T4 after skin incision, T5 after chest closure and T6 after extubation were lower than those in single group and control group.

## 4. Discussion

The outcome of this research implies that SAPB with Nalbuphine is essential in minimizing initial pain of post operation after the lung resection of VATS with minimal side effects. This study has been critical in analyzing the effective outcomes of SAPB in randomized regulated attempts or trials after thoracoscopic surgery for postoperative Nalbuphine [7]. This research proved significance in demonstrating that there was no major difference in the scores of VAS score between the placebo group and the SAPB group during the initial 24 hours after the process of operation. Concurring with Piccioni et al [8], there was efficacy of the SAPB when it came to the postoperative reprieve of the chest walls of the elderly patients as the medicinal doses of Nalbuphine in the SAPB set or group were marginally lower, and the time required to utilize the first doses of Nalbuphine was palpably longer [9]. The research judging from the results was significant in attesting the efficacy of SAPB in reducing postoperative pain around the chest wall whilst minimizing the postoperative prescription of opioids [10]. The overriding difference is that VATS does not function effectively as SAPB when it comes to minimizing postoperative pain [11].

From this research study, there was contrast in that local infiltration Nalbuphine and SAPB for postoperative analgesia after the VATS established that elderly people in the SAPB group possessed superior VAS scores during the initial 8 hours postoperatively; this is despite the dosage of Nalbuphine being significantly lower. Chen et al [12], avers that a preliminary meta-analysis on the Nalbuphine result of SAPB in elderly people going through thoracoscopic surgery demonstrates that Nalbuphine amalgamated with SAPB minimizes the perioperative chest pains among the elderly patients. This is particularly when compared to the VATS treatment. Centered from the results of this research, the Nalbuphine score on the SAPB group at 6-, 12- and 24 hours after the thoracoscopic surgery was lower compared to that of the control set. This proves that that Nalbuphine treatment has better efficacy levels at 6 hours compared to when it was at 24 hours.

Deng et al [13] asserts the period to the VAS score four after the process of operation was considerably reduced, (median 12 hours) in the control group versus the SAPB group. This ostensibly shows that the number of elderly patients necessitating advance Nalbuphine during the initial twelve hours after the process of operation was considerably lower. Moreover, there are similarities both at home and abroad in that SAPB is effective compared to local infiltration at the site of incision for postoperative management of chest pains among the elderly patients after VATS resection of the lung [14]. The difference is that period of Nalbuphine abroad in our SAPB group surpassed the initial levels suggesting that higher concentrations of Nalbuphine were used [15].

The article "Effects of Nalbuphine Combined with Anterior Serratus Plane Block in Elderly Patients Undergoing Thoracoscopic Surgery" was published in 2022. Journal: J Healthc Eng.

Initially, even though local Nalbuphine or nerve block, among the elderly patients was not done in the presence of the surgical anesthetists and operating surgeons, the anterior serratus plane block method was arbitrated in accordance with the needle puncture mark [16]. Nonetheless, the surgeons adjusted the Nalbuphine centered on PTi monitoring and sedation threshold index that has minimal effect on the management of opioids and Nalbuphine depth [17]. The other significant difference is severity and presence of pain by elderly patients suffering cognitive disorders. Hence, over the years, there has been more and more objective assessment techniques. Nalbuphine not only considerably constrains the actions of the cerebral cortex but also maintains integral the actions of the subcortical autonomic nervous system among the elderly patients. As attested through this research when undergoing thoracoscopic surgery, the major signs that damages the stimuli might encompass variations such as diaphoresis, pulse wave amplitude, pupil diameter, blood pressure, and increased heart rate among the elderly people [18]. The entirety of this condition is because of changes or suppression when it comes to the balance of parasympathetic and sympathetic nerve actions. The present study did not have the comparison on the analog pain notch due to lack of the data. The future studies should perform the analysis on this topic.

## 5. Conclusion

In conclusion, SAPB combined with Nalbuphine is a convenient and safe regional nerve block method for VATS, which in effect alleviates initial wound pain among the elderly, offers protracted-lasting analgesia compared to local infiltration at the incision, and constrains the requirement for initial postoperative advance Nalbuphine.

## Figures and Tables

**Figure 1:** The flow chart of the study.

**Table 1:** Comparing the Overall Medical Data among Two Group

Group	N	Female/male	Age (Years)(Mean ± SD)	BMI (kg/m2) (Mean ± SD)	Operation Time (min) (Mean ± SD)
Control	30	13/17	58.21 ± 9.02	23.84 ± 2.94	98.22 ± 27.87
SAPB	30	15/15	56.21 ± 7.21	24.46 ± 2.86	107.70 ± 27.15
Nalbuphine	30	12/18	57.90 ± 7.38	23.59 ± 2.61	98.43 ± 28.24
Nalbuphine + SAPB	30	14/16	57.83 ± 8.22	23.27 ± 2.94	99.37 ± 29.16
P value		0.540	0.295	0.392	0.219

The article "Effects of Nalbuphine Combined with Anterior Serratus Plane Block in Elderly Patients Undergoing Thoracoscopic Surgery" was published in 2022. Journal: J Healthc Eng.

**Table 2:** Number of Patients Needing Extra Nalbuphine at Different Time Points after Surgery

Group	6 hours	12 hours	24hours	48 hours
Control	11	15	3	1
SAPB	9	13	3	2
Nalbuphine	8	11	3	2
Nalbuphine + SAPB	4	6	2	1
P value	0.028	0.037	1.00	1.00

**Table 3:** Propofol Dose and Intraoperative Remifentanil (mean ± SD)

Group	N	Intraoperative Remifentanil Dose Operation (ug)	Intraoperative Propofol Dose (mg)
Control	30	242.66 ± 97.42	763.24 ± 102.71
SAPB	30	250.88 ± 66.84	748.68 ± 72.61
Nalbuphine	30	248.62 ± 48.39	757.53 ± 81.59
Nalbuphine + SAPB	30	251.57 ± 73.76	752.41 ± 89.26
P value		0.659	0.427

**Table 4:** Adverse Responses

Group	Vomiting and Nausea
Control	3 (10%)
SAPB	4 (13%)
Nalbuphine	3 (10%)
Nalbuphine + SAPB	2 (7%)
P value	1.00

**Table 5:** The comparison for the postoperative recovery.

Group	Spontaneous respiratory recovery time (hours)	Extubation time (hours)	Resuscitation room stay time (hours)	Incidence of extubation cough	Restlessness and respiratory depression
Control	0.88 ± 0.11	1.92 ± 0.13	6.5 ± 1.2	4	5
SAPB	0.78 ± 0.24	1.77 ± 0.55	5.9 ± 2.2	4	4
Nalbuphine	0.69 ± 0.11	1.85 ± 0.42	7.1 ± 1.1	5	3
Nalbuphine + SAPB	0.55 ± 0.05	1.1 ± 0.11	4.1 ± 1.6	1	1
P value	<0.05	<0.05	<0.05	<0.05	<0.05

## Data Availability

The simulation experimentation data utilized to back the conclusions of this research are accessible from the agreeing writer upon demand.
